The article "Ultrasound of Fetal Cardiac Function Changes in Pregnancy-Induced Hypertension Syndrome" was retracted in 2023. Reasons: unreliable results or conclusions; concerns about the data; concerns about the peer review; concerns about the citations.

# Ultrasound of Fetal Cardiac Function Changes in Pregnancy-Induced Hypertension Syndrome

**DOI:** 10.1155/2022/2019869

**Published:** 2022-04-27

**Authors:** Maoting Lv, Shanshan Yu, Yongzhen Li, Xiaoting Zhang, Dan Zhao

**Affiliations:** ^1^Second Department of Ultrasound Diagnosis, Cangzhou Central Hospital, Cangzhou, China; ^2^Delivery Room, Cangzhou Central Hospital, Cangzhou, China; ^3^Second Department of Neurosurgery, Cangzhou Central Hospital, Cangzhou, China

## Abstract

Pregnancy-induced hypertension syndrome (PIH) is a common pregnancy syndrome that could cause varying degrees of maternal and fetal organic damage and even endanger their lives. This study aimed to investigate ultrasound of fetal cardiac function changes in PIH. Totally 40 cases of gestational hypertension admitted to Cangzhou Central Hospital between October 2018 and September 2019 were enrolled in the hypertension group, and 40 women with healthy pregnancies during the same period were assigned to the normal group. Ultrasound results showed that PIH was associated with a significantly higher fetal cardiac septal thickness, fetal left ventricular end-diastolic area and end-systolic area, fetal right ventricular end-diastolic area and end-systolic area, fetal left ventricular systolic fraction 1 (VSF1), fetal left ventricular systolic fraction 2 (VSF2), fetal right VSF1, and fetal right VSF2 versus healthy pregnancy. The PIH fetuses had significantly lower neonatal weights versus healthy fetuses. Newborns of hypertensive pregnancies have larger hearts, faster heart rates, increased cardiac contractility, and lower weights versus newborns of healthy pregnancies.

## 1. Introduction

Pregnancy-induced hypertension syndrome (PIH) is a common pregnancy syndrome that could cause varying degrees of maternal and fetal organic damage and even endanger their lives [1, 2]. Its development is mostly seen after 20 weeks of gestation and is characterized by hypertension and other systemic dysfunctions, with a prevalence of 5%. PIH is potentially associated with generalized edema, nausea, vomiting, headache, blurred vision, epigastric pain, thrombocytopenia, coagulation dysfunction, fetal growth retardation, or even maternal and fetal death in severe cases [3]. Moreover, it also features a high risk of miscarriage, intrauterine growth retardation, and perinatal mortality when compared with normal pregnancies [4, 5].

Due to the unknown etiology of PIH, the treatment mostly relies on spasm lysis, hypotension, diuresis, and timely termination of pregnancy according to its predisposition factors and pathophysiological changes. This disease seriously compromises maternal and child health and is one of the leading causes of morbidity and mortality in pregnant women and perinatal children. Therefore, early detection and assessment of fetal cardiac function are paramount to guide clinical assessment of the condition for further treatment [6]. Echocardiography is a common modality for the structural and functional examination of the heart, with simple operation and good repeatability, which allows an efficient assessment of the fetal cardiac function and provides a reference basis for early detection of cardiac developmental abnormalities [7, 8]. Previous research has confirmed that color Doppler ultrasound techniques can evaluate the hemodynamics of fetuses with higher sensitivity and accuracy and is considered an optimal method for fetal hemodynamics monitoring [9].

The article "Ultrasound of Fetal Cardiac Function Changes in Pregnancy-Induced Hypertension Syndrome" was retracted in 2023. Reasons: unreliable results or conclusions; concerns about the data; concerns about the peer review; concerns about the citations.

The present study was conducted to compare the cardiac function of fetuses of PIH with those of normal pregnancy through ultrasound to investigate the diagnostic value of ultrasound for PIH on fetal cardiac function changes and its significance for clinical reference.

## 2. Materials and Methods

### 2.1. Baseline Data

Between October 2018 and September 2019, 40 cases of PIH admitted to our institution were assessed for eligibility and recruited in the hypertension group, and 40 women with healthy pregnancies during the same period were assigned to the normal group. All 80 cases in both groups were singleton fetuses with no malformations after examinations. The study was ethically approved by the Ethics Committee of Cangzhou Central Hospital (2018-JY225).

### 2.2. Inclusion and Exclusion Criteria

#### 2.2.1. Inclusion Criteria

It includes (a) patients with singleton pregnancies; (b) patients with PIH who met the diagnostic criteria of the syndrome in the hypertension group; (c) patients with normal communication skills; and (d) patients with knowledge and consent to the study content.

#### 2.2.2. Exclusion Criteria

It includes (a) patients with fetal malformations; (b) patients with fetuses with congenital heart disease; and (c) patients with abnormal liver and kidney functions.

### 2.3. Methods

#### 2.3.1. Routine Examination

Fetal biparietal diameter, head perimeter, femoral length, amniotic fluid index, and placenta condition were measured.

#### 2.3.2. Fetal Examination

The fetal spine, liver, and gastric vesicles were identified as the left and right ventricles of the heart. The thickness of the diastolic interventricular septum (IVS) was measured under a four-chamber heart view. The left ventricular end-systolic perimeter and area (LVSP, LVSA), right ventricular end-systolic perimeter and area (RVSP, RVSA), and right and left ventricular end-diastolic perimeter and area (LVDP, LVDA, RVDP, RVDA) were measured as per the different phases of the heart and playback function.

The article "Ultrasound of Fetal Cardiac Function Changes in Pregnancy-Induced Hypertension Syndrome" was retracted in 2023. Reasons: unreliable results or conclusions; concerns about the data; concerns about the peer review; concerns about the citations.

#### 2.3.3. Calculation of Ventricular Systolic Fraction

Ventricular systolic fraction 1 (VSF1) = (ventricular end-diastolic perimeter−ventricular end-systolic perimeter)/ventricular end-diastolic perimeter. Ventricular systolic fraction 2 (VSF2) = (ventricular end-diastolic area−ventricular end-systolic area)/ventricular end-diastolic area.

### 2.4. Statistical Analysis

SPSS 20.0 was used for data analyses, and GraphPad Prism 8 was used for image rendering. The measurement data were expressed as ($\bar{x}$ ± *s*) and processed using independent samples *t*-test. The count data were expressed as (*n*, %) and analyzed using the chi-square test. Differences were considered statistically significant at *P* < 0.05.

## 3. Results

### 3.1. General Data of the Pregnant Women

The baseline data of the hypertension group (aged 23–36 years, mean age of [28.57 ± 3.46] years, 24–33 weeks of gestation, mean gestational week of [28.43 ± 3.74], gravidity of 1–3 times, mean gravidity of [1.27 ± 0.44] times) were comparable with those of the normal group (aged 23–35 years, mean age of [28.17 ± 3.35] years, 24–33 weeks of gestation, mean gestational week of [28.61 ± 3.52], gravidity of 1–3 times, mean gravidity of [1.25 ± 0.47] times) (*P* > 0.05) (Table 1).

### 3.2. Morphological Changes of the Fetal Heart

The fetal ventricular perimeter and area in systole and diastole and the thickness of the ventricular septum were significantly greater in the hypertension group than in the normal group (*P* < 0.05). PIH exerts a greater effect on the right cardiac system than on the left cardiac system (Table 2).

### 3.3. Ultrasound Changes of Fetal Heart Function

In the hypertension group, the FVSF1 was (0.24 ± 0.09), the FVSF2 was (0.38 ± 0.15), the RVSF1 was (0.24 ± 0.03), and the RVFS2 was (0.35 ± 0.08), while the above indicators were (0.13 ± 0.04), (0.20 ± 0.09), (0.16 ± 0.10), and (0.21 ± 0.14) in the normal group. The systolic fractions of both the left and right ventricles were significantly higher in the fetuses of the hypertension group versus those of the normal group (*P* < 0.05) (Table 3).

### 3.4. Comparison of Neonatal Weight

The weight of the newborns in the hypertension group was (3036 ± 761) *g* and that of the newborns in the normal group was (3486 ± 589) *g*. PIH newborns showed significantly lower neonatal weights versus healthy newborns (*P* < 0.05) (Figure 1).

## 4. Discussion

The results of the present study showed a significantly higher fetal ventricular systolic and diastolic perimeter and area and septal thickness in the hypertension group than in the normal group, which indicates that maternal hypertension in pregnancy may seriously compromise the fetal cardiac function. Meanwhile, PIH causes a greater impact on the fetal right heart system than the left heart system, suggesting a larger right heart system than the left heart system in fetuses of PIH [10, 11]. In addition, the systolic fractions of both the left and right ventricles of the fetuses in the hypertension group were significantly higher than those of the fetuses in the normal group, suggesting that PIH patients are associated with varying degrees of impact on fetal cardiac function, which may presumably be attributed to the early changes in blood flow in patients with PIH, hypercoagulability of the blood, increased viscosity of the blood, and spasm of the small arteries throughout the patient's body, leading to impaired cardiac function in both the mother and the fetus [12]. Furthermore, the hypertension group had significantly lower neonatal weights versus the normal group, which may be attributable to the constriction and narrowing of the spiral artery and the target vessel of the placenta, resulting in the reduction of blood flow in the small spiral arteries of the meconium layer, ischemia, and hypoxia in the intervillous space and small vessels of the meconium, thereby compromising the growth and development of the fetus and causing fetal weight loss [13, 14]. Sound maternal health care, proper diet, and maintenance of a positive psychological state can prevent the development of PIH in pregnant women to achieve timely and accurate judgment, prevention, and aggressive treatment, which are considered effective in reducing maternal and infant morbidity and mortality [15].

The article "Ultrasound of Fetal Cardiac Function Changes in Pregnancy-Induced Hypertension Syndrome" was retracted in 2023. Reasons: unreliable results or conclusions; concerns about the data; concerns about the peer review; concerns about the citations.

PIH is a syndrome specific to pregnant women [16, 17] and may trigger systemic small artery spasm in patients, leading to increased peripheral vascular resistance and consequently placental dysfunction [18, 19]. In the case of ischemia and hypoxia, the compensatory function initiated by the fetal organism is associated with redistribution of fetal cardiac output, compensatory hypertrophy of cardiomyocytes, and impairment of cardiac diastolic and systolic function. Thus, early and accurate assessment of fetal cardiac function in patients with PIH is essential for the health of the mother and the fetus. The ultrasound features of the sonogram of the PIH fetus depend on the conditions of the pregnant patients, namely, a normal fetal sonogram for short disease duration and mild condition, and a fetal intrauterine growth retardation sonogram for long disease duration and severe condition [20, 21]. The function of the primitive fetal heart appears approximately 21 d after fertilization. The current resolution of ultrasound apparatus enables the detection of fetal heart activity at the 6th week of gestation, with a flicker-like beating performance at a faster frequency, while the absence of fetal heart activity at the 8th week of gestation indicates abnormalities. Fetal movement is the movement of the fetal body in the amniotic fluid and can be detected slightly later than the fetal heart activity, and a reliable fetal movement detection requires an absolute still of the pregnant woman's body position, the examination bed, and the probe site.

The article "Ultrasound of Fetal Cardiac Function Changes in Pregnancy-Induced Hypertension Syndrome" was retracted in 2023. Reasons: unreliable results or conclusions; concerns about the data; concerns about the peer review; concerns about the citations.

## 5. Conclusion

The PIH fetuses had significantly lower neonatal weights versus healthy fetuses. Newborns of hypertensive pregnancies have larger hearts, faster heart rates, increased cardiac contractility, and lower weights versus newborns of healthy pregnancies.

## Figures and Tables

**Figure 1:** Comparison of neonatal weight. Note: # indicates P <0.05.

**Table 1:** Comparison of baseline data ($\bar{x}$ ± s).

	Hypertension group (*n* = 40)	Normal group (*n* = 40)	*t*	*P* value
Mean age	28.57 ± 3.46	28.17 ± 3.35	0.525	0.601
Mean gestational weeks	28.43 ± 3.74	28.61 ± 3.52	−0.222	0.825
Gravidity	1.27 ± 0.44	1.25 ± 0.47	0.196	0.845

**Table 2:** Morphological changes of the fetal heart ($\bar{x}$ ± *s*).

	Hypertension group (*n* = 40)	Normal group (*n* = 40)	*t*	*P* value
IVS (mm)	5.71 ± 0.92	4.07 ± 0.77	8.646	<0.001
LVDP (mm)	69.35 ± 8.41	60.44 ± 6.33	5.354	<0.001
LVSP (mm)	55.28 ± 8.13	48.37 ± 6.02	4.32	<0.001
LVDD (cm^2^)	3.51 ± 0.98	2.36 ± 0.85	5.607	<0.001
LVSD (cm^2^)	2.43 ± 0.72	1.91 ± 0.67	3.344	0.001
RVDP (mm)	71.84 ± 7.98	58.43 ± 5.88	8.556	<0.001
RVSP (mm)	63.47 ± 8.56	55.49 ± 7.43	4.453	<0.001
RVDD (cm^2^)	3.66 ± 0.82	3.15 ± 0.61	3.156	0.002
RVSD (cm^2^)	2.87 ± 0.80	2.13 ± 0.64	4.568	<0.001

**Table 3:** Ultrasound changes of fetal heart function ($\bar{x}$ ± *s*).

	Hypertension group (*n* = 40)	Normal group (*n* = 40)	*t*	*P* value
FVSF1	0.24 ± 0.09	0.13 ± 0.04	7.064	<0.001
FVSF2	0.38 ± 0.15	0.20 ± 0.09	6.508	<0.001
RVSF1	0.24 ± 0.03	0.16 ± 0.10	4.846	<0.001
RVFS2	0.35 ± 0.08	0.21 ± 0.14	5.491	<0.001

## Data Availability

The datasets used during the present study are available from the corresponding author upon reasonable request.
